The article "Early Stroke Prediction Methods for Prevention of Strokes" was retracted in 2023. Reasons: signs of a paper mill; suspected computer-generated content; unreliable results or conclusions; concerns about the data.

# Early Stroke Prediction Methods for Prevention of Strokes

**DOI:** 10.1155/2022/7725597

**Published:** 2022-04-11

**Authors:** Mandeep Kaur, Sachin R. Sakhare, Kirti Wanjale, Farzana Akter

**Affiliations:** ^1^Department of Computer Science, Savitribai Phule Pune University, Pune, India; ^2^Computer Engineering Department, Vishwakarma Institute of Information Technology, Kondhwa (Bk), Pune, India; ^3^Department of ICT, Bangabandhu Sheikh Mujibur Rahman Digital University, Bangladesh

## Abstract

The emergence of the latest technologies gives rise to the usage of noninvasive techniques for assisting health-care systems. Amongst the four major cardiovascular diseases, stroke is one of the most dangerous and life-threatening disease, but the life of a patient can be saved if the stroke is detected during early stage. The literature reveals that the patients always experience ministrokes which are also known as transient ischemic attacks (TIA) before experiencing the actual attack of the stroke. Most of the literature work is based on the MRI and CT scan images for classifying the cardiovascular diseases including a stroke which is an expensive approach for diagnosis of early strokes. In India where cases of strokes are rising, there is a need to explore noninvasive cheap methods for the diagnosis of early strokes. Hence, this problem has motivated us to conduct the study presented in this paper. A noninvasive approach for the early diagnosis of the strokes is proposed. The cascaded prediction algorithms are time-consuming in producing the results and cannot work on the raw data and without making use of the properties of EEG. Therefore, the objective of this paper is to devise mechanisms to forecast strokes on the basis of processed EEG data. This paper is proposing time series-based approaches such as LSTM, biLSTM, GRU, and FFNN that can handle time series-based predictions to make useful decisions. The experimental research outcome reveals that all the algorithms taken up for the research study perform well on the prediction problem of early stroke detection, but GRU performs the best with 95.6% accuracy, whereas biLSTM gives 91% accuracy and LSTM gives 87% accuracy and FFNN gives 83% accuracy. The experimental outcome is able to measure the brain waves to predict the signs of strokes. The findings can certainly assist the physicians to detect the stroke at early stages to save the lives of the patients.

## 1. Introduction

Nowadays, due to technological advancements, life expectancy of human being is rising day by day. The lifestyle has been changed from active lifestyle to sedentary lifestyle due to the advent of technical gadgets such as laptops, smart phones, and portable devices. Not only the aging society but the young generation is also facing many health problems such as cardiovascular diseases, diabetes, hypertension, and strokes due to inactive lifestyle. There is a need of smart health-care devices to monitor the health of individuals by using some biomarkers and noninvasive smart techniques. The studies in the exiting literature produce evidences of bad impact of sedentary lifestyle on human health [1–3]. In this paper, we are focusing on the problem of strokes, and an attempt is made to devise a system which uses bioelectrical images to predict the strokes. The major cause behind stroke is disruption of blood supply due to clotting in the blood to the nerves in the brain. The stroke can be major or minor. In minor stroke, the blood supply to some parts of the brain is hampered, and in major stroke, the person can lose life. Stroke is an emergency health condition which has to be dealt with carefully. The common symptoms include trouble in movement, confusions, improper verbal communication, and difficulty in understanding. Stroke causes long-term neurological damage and death.

There are two categories of stroke, ischemic embolic and hemorrhagic. Ischemic embolic stroke occurs when there is a blood lump at heart and not in the brain, and it narrows the brain arteries. In hemorrhagic stroke, there is blood leakage at the artery in the brain due to the damage. For elderly generation, stroke can be lethal. The heart gets damage during the heart attack and stroke damage the brain in a similar manner. Once a person is diagnosed with stroke disease, it needs continuous health monitoring. The stroke starts with a ministroke which is known as transient ischemic attacks (TIA). It is the condition which reveals that the person will face stroke within a couple of days from the occurrence of the ministroke. The World Health Organization (WHO) claims that there are frequent deaths due to stroke [4]. If stroke is detected or diagnosed early, the loss of death and severe damage to brain can be prevented in 85% cases [5]. Extra care is needed for senior citizens as it is more lethal for the aging community. A disease like stroke needs continuous monitoring and observation. The rate of stroke cases is increasing day by day due to stress, inactivity, consumption of drugs, and bad dietary habits [6].

Stroke causes dysfunctionalities at some parts of the brain locations which results into problems in the brain blood vessels [6]. In 2016, WHO has published one report which reveals that stroke is the second most growing reason of disability in the current population worldwide. In the past 40 years, it has been observed that the number of cases of stroke doubled with the passage of each decade [7]. There is no specific treatment in medical science for handling strokes; therefore, early diagnosis is the key to handle strokes. The early detection can prevent disabilities, loss of deaths, and other brain-related severe ailments [8]. In most of the stroke identification-existing studies, magnetic resonance imaging (MRI) and computed tomography (CT) are used, but these techniques expose the patients to radiations or probable allergic reactions. Secondly, MRI or CT scans are very expensive methods for diagnosis, and people in underdeveloped countries cannot take advantage of these techniques due to excessive cost. Nowadays, noninvasive techniques such as EEG (electroencephalogram) are getting popularity which is also cost-effective or nonexpensive technique [9, 10]. COVID-19 has also increased the cases of strokes. Many authors have investigated the correlation between the history of strokes and deaths of the hospitalized patients with COVID-19 [4]. From the comprehensive study of 3248 patients, it is found that history of stroke is significantly associated with the deaths of hospitalized patients. The clinical course of COVID-19 patients with the history of stroke is examined. Even in COVID-19 patients, the noninvasive techniques have played a great role in identification of strokes. The studies are also correlating stress and depression with strokes [11].

### 1.1. Related Work

This subsection discusses the exiting works in the area of the proposed research.

The study presented in [6] is also devising a software-based model where screening of depression is performed with deep learning and EEG signals are used to distinguish between normal brain signals and abnormal brain signals which induce strokes. The authors also found that right hemisphere signals are more idiosyncratic during depression as compared to the left hemisphere. In [12], the authors have invented one device for detection of stroke along with time and duration. In [7], the authors have combined EEG with galvanic skin response (GSR) signals for the diagnosis of strokes, but the accuracy is 73.8%. In [9], the authors have used EEG data without using the frequency characteristics of EEG. Real-time data is gathered from EEG sensors to develop and train the stroke detection model. In [10], the authors have combined the bioelectrical signals with natural language processing, and then, machine learning is used for classification of strokes and normal signals. In [11], a bidirectional deep neural network is used for EEG-based image classification. The information of signals is processed at various regions to distinguish between right and left hemispheres of the brain. Finally, the classification is made between abnormal and normal signals. Paper [13] uses sparse representation (SR) and CNN for classification of MRI images to detect strokes. In [14], the deep learning-based classification is utilized that learns from end-to-end information without extracting handcrafted features and considers multiple bioelectrical signals for classification.

In [15], the authors have used time series concept for classification of brain signals by transforming single-dimensional time series to a double-dimensional image classification problem. In [16], the authors have devised a prediction model that shows stepwise improvement in the correct prediction of brain signals to detect the early stages of strokes. In article [17], the authors have utilized EEG signal-based classification, and prior to applying classification techniques, the signals are transformed into images, and then, neural networks are applied for detection of strokes. The aim of [18] is to use deep neural network for decoding the EEG signals. The authors have examined the methods for single-trial and multitrial EEG classification. The researchers have proposed many approaches [19–23] for dealing with strokes to minimize the damage of brain tissues. The existing techniques have certain flaws such as time complexity for producing the results, expensive data generated by using MRI or CT scans, and space complexity where finding solution is difficult to determine the difference between ministroke (TIA) and actual stroke. In order to overcome these problems, this paper is proposing a noninvasive technique for identifying the bioelectrical signals (specifically EEG) with deep learning models to predict the strokes at early stage.

The highlights of the stroke prediction strategy are as follows:

- The strategy is using deep learning-based predictors to predict the strokes. Three deep learning models are devised to test the efficacy of three different models because accurate prediction plays important role in predicting the results
- The first phase collects the raw data based on EEG bioelectrical signals
- The next phase extracts the features from the data and the characteristics of the frequency of signals
- The stored signal-based data is consumed as an input to the deep learning-based modules
- Then, the time series-based prediction module is invoked which predicts whether the patient can have stroke or TIA
- The predicted stroke outputs are compared with the actual outputs to judge the efficacy of the time series-based deep learning models

The paper is organized into four sections. The next section highlights the methods used in the research study. The results and inferences are presented in the third section of the paper. The last part is summarizing the paper work.

## 2. Proposed Methods

The methods proposed in this paper are based on time series prediction methods. The steps of the proposed method are described below and also shown in Figure 1.

- The first phase collects the raw data based on EEG bioelectrical signals
- The next phase extracts the features and the important characteristics of the frequency of signals
- The next phase prepares the model based on deep learning-based predictors
- The stored signal-based data is consumed as an input to the deep learning-based modules
- Then, the time series-based prediction module is invoked which predicts whether the patient can have stroke or TIA

### 2.1. Collection of Bioelectrical Signals (EEG, ECG, and EMG) through Smart Sensing Devices

The bioelectrical signals such as EEG (electroencephalography) are collected through sensors as in our research work. We have made use of noninvasive technique. EEG is preferred over other two techniques, ECG (electrocardiography) and EMG (electromyography), as other methods are invasive methods. The easiest method is adopted to collect the RAW data as bioelectrical signals. The bioelectrical signals can help in diagnosis of strokes as the sequence of signals reveal whether everything is normal or there are some abnormalities in terms of TIA or strokes.  Figure 2 is depicting the bioelectrical signal-based collection of data where brain signals are recorded to reveal the conditions of strokes in earlier stages.

### 2.2. Porting of RAW Data to the Server

The EEG data is gathered by using six channels at predetermined frequency of 1000 Hz. The data is collected in the form of bioelectrical signals, and the collected data is ported to the server. The server prepares the database of the collected raw data. The data is then prepared for preprocessing, and then, the features are extracted. The signals of EEG are categorized into five types of signals as shown in Figure 3. The categories include alpha, beta, gamma, theta and delta. It is very important to use these categories of the signals to detect normal people and stroke affected people.

### 2.3. Stroke Forecasting Module

The next is our stroke forecasting module which is based on deep neural networking techniques. The series of processes contribute in this module where we have taken up four algorithms for checking the viability of the algorithms on the problem statement of detection of early strokes. The first algorithm is FFNN which is feeding the neural network in a forward manner, the next is LSTM (a better version of recurrent neural network), an attempt is made to try with bidirectional LSTM (biLSTM), and then finally, GRU has been tried to produce the more accurate results. The deep learning methods get the input as raw data of EEG signals, the waveline analysis is learned from an offline data, and then, the trained algorithms are tried on the actual data to analyze the wave signals. In order to learn from the offline data, the neural networks are trained against all types of possible signals of brain to identify strokes. Since the patterns are almost fixed and almost all the signals find their similar signals in the offline dataset for training, the testing results are quite promising. The trained and tuned module can certainly predict whether the signals belong to a person who is having stroke or to a normal person.

The LSTM algorithm forecasts the next stage by keeping historical and futuristic information as LSTM has forget gates to remember more data. The biLSTM overcomes the shortcomings of LSTM by incorporating a backward processing layer in normal LSTM. The biLSTM is more powerful than LSTM in providing accuracy as biLSTM can infer from the historical data for the future and also perform the reverse inference from future to history. The GRU is also tried as GRU is less complex and delivers the results in lesser span of time. While LSTM has three gates, GRU has two gates, reset and update. Feed forward is also tried with the EEG data to make the comparison of the deep learning techniques and to evaluate the output accuracy.

#### 2.3.1. Prediction Framework

To predict the early strokes on the basis of symptoms recorded in terms of data fields, the neural network-based predictors are proposed as transfer learning models which learn from the offline data and can be applied on the online quick data for predicting the likely chances of strokes. The predictors are designed into threefold strategy: Processing of data during training, to train the model from offline stroke-based data, and transfer phase where offline training is applied on online data for prediction of strokes.

*(1) Data Processing*. The data has to be processed after receiving the offline data to train the stroke prediction model, and when the data is collected online, then the collected data is transformed in discrete units. The discrete units are then supplied to the predictor in a sequence.

*(2) Module Preparation*. The stroke predictor requires building of the model based on the input data, and this phase is very important; the second phase is of prime importance which builds the model. We have adopted three-layered structures to minimize the time complexity and to keep the model simple for usage of physicians. Layer one is the input layer, and it contains neurons which represents dimension of the stroke-based data. The hidden or intermediate layer is decided by the empirical study to get the more accurate results. The output layer predicts whether the patient can have strokes or not.

*(3) Training Phase*. The training phase begins with the module training on offline stroke-based data. This phase optimizes the loss function value to retain the information intact between the layers and to help the model to converge at global optima solution. In biLSTM and GRU, ion filter is adopted to escape the model from converging at local optima.

*(4) Testing Phase*. The predictors are tested on the online or real-time data to check the efficacy of the models. It is found that GRU-based predictor gives the most accurate stroke prediction results, followed by biLSTM and FFNN methods.

#### 2.3.2. Analysis of the Outcome

Once the output is received from the proposed methods, the outcome is evaluated against the statistical performance evaluators to check whether the proposed algorithms are predicting with accuracy whether the person is normal or can have ministroke (TIA) or actual stroke. The analysis is made on the basis of RMSE score (root mean square error), MAE (mean absolute error), MSE (mean squared error), MRE (mean relative error), and time consumption for producing output.

#### 2.3.3. GUI-Based Output

The final module is graphically presenting the results to the user whether the input data shows abnormality in the wavelines and a person can experience stroke in the near future or everything is normal.

## 3. Results and Inferences

### 3.1. Experimental Results

In this subsection, the performance is evaluated on the basis of statistical metrics. We have used statistical error analysis to predict the capability of proposed techniques. To evaluate the prediction capability of the proposed GRU, biLSTM, and other prediction methods, the statistical error analysis methods are used. In order to obtain the results, the machines with special configuration capabilities are used to train the models such as 16 GB RAM, GPU—NVIDIA GeForce GTX 940, and Microsoft Windows 10 (64-bit) platform. GPUs are required to train the deep neural networks, and after training, testing is also performed on the same machines.

1. Mean absolute error (MAE) represents median of all the absolute errors and formulae is expressed below in Equation (1).

(1) $$\begin{array}{c} \text{MAE}=\frac{1}{m}\overset{m}{\underset{a=1}{\sum }}\left|X_{a}-X\right|, \end{array}$$

where the number of errors is represented by *m*, *∑* represents addition of all values, and |*X*_*a*_ − *X*| is the absolute errors

In the following chart (Figure 4), the mean absolute error value for each technique is displayed. It is obtained for all the prediction methods (GRU, biLSTM, LSTM, and FFNN) reflected in the proposed work section. The results demonstrate that for proposed GRU method has achieved highest accuracy with minimal error, the MAE score for biLSTM is also better than other techniques considered in the study such as LSTM and FFNN. It is found that biLSTM is performing far better than the conventional LSTM as it has ability to work in a forward as we all backward direction. The feed forward method is not performing well in the time series problem.

(2) Root mean square error (RMSE) depicts the standard deviation of the predicted errors. The formula for it is expressed in Equation (2).

(2) $$\begin{array}{c} \text{RMSE}=\sqrt{\frac{\sum_{a=1}^{m}{\left(X_{a}-{\overset{\wedge }{X}}_{a}\right)}^{2}}{M},} \end{array}$$

where *M* is equal to the number of nonmissing data points, *a* is the variable, *X*_*a*_ is the actual observations of time series and ${\hat{X}}_{a}$ represents forecasted time series

In the chart (Figure 5), RMSE values are presented for all the applied algorithms. Proposed GRU algorithm gives excellent results with respect to RMSE score and beats other algorithms considered for study.

(3) Mean squared error (MSE) is a summary of the prediction ability and accuracy predicted for the proposed GRU model. A formula for it is given in Equation (3).

(3) $$\begin{array}{c} \text{MSE}=\frac{1}{m}*\sum {\left(\text{actual}-\text{predicted}\right)}^{2} \end{array}$$

The results of MSE scores are given in Figure 6. It can be inferred that GRU gives the best accuracy, followed by biLSTM, LSTM, and FFNN. In this paper, we have compared proposed GRU*-*based prediction algorithm with three comparative algorithms which are benchmarked methods for the prediction of the stroke. When we compare GRU with the LSTM and FFNN stroke prediction algorithm, performance of the GRU is best. It also has ability to predict by retaining relevant information in its layers. The biLSTM is capable to process short-term time series, whereas GRU can consider long-term series also. It is observed from statistical continuity that LSTM does not support nonlinear fitting capability. Performance of the LSTM is good in the diagnosis of strokes diseases, but sometimes, the relevant information is lost in the hidden layers. Accuracy of GRU is more as compared to LSTM.

To verify the time complexity and efficiency of convergence of the algorithms, the iterations for training set are defined similarly for the algorithms considered for the research, and it is observed from Figure 7 that the GRU outperforms other techniques with respect to MRE scores. However, the beginning relative error of the proposed GRU is higher, and gradually, it decreases. The other techniques also behave in the same manner, but GRU shows the best performance with respect to the MRE scores.

(4) Specificity and sensitivity scores are used to measure the accuracy in the results produced by the implemented algorithms

Figure 8 demonstrates the sensitivity and specificity scores obtained by the various methods. All the methods work well for classifying the strokes, but the proposed GRU stroke identification or forecasting method outperforms other forecasting models. The time series-based models, LSTM and biLSTM, also perform well and provide quite accurate results. Timely forecasting is very important to save the life of the patient. Delay in prediction may lead to fatal outcomes. The specificity allows the correct identification of patients who can have strokes in the near future. The sensitivity specifies how often the proposed forecasting models can correctly generate the positive results for the patients who can definitely have problem of strokes in the near future.

### 3.2. Analysis

Stroke is related to the serious brain condition which can give rise to severe problems like reduction in blood perfusion, decrease in glucose supply, and decrease in oxygen supply in the brain. It may lead to paralysis attack or may lead to death as well. The brain's electrical activity in case of ischemic stroke is associated with hypoperfusion of cerebral tissues. An ischemic stroke is a serious condition which hampers the blood supply to the brain, and it prevents the tissues of the brain from getting enough oxygen for proper functioning of the brain. In this case, brain cells start dying in minutes. The hemorrhagic stroke occurs due to a burst or permeable blood vessels that bleed into the brain. The reduction in blood supply to the brain damages tissues and causes paralysis, numbness in arm, face, or leg, slurred speech, behaviour changes, loss of balance, dizziness, nausea, or severe headache. The damage caused by stroke is irreversible. Hence, this paper attempts to bring a solution in the form of early stroke prediction model which can reveal whether the person can have stroke in the future on the basis of biomarkers study, EEG signals, and the characteristics of the frequency of signals. We have made use of deep learning models in this research study for accurate predictions of the early stroke conditions. The four deep learning models are tried, and their respective results are compared in this section to judge the accuracy and viability of the proposed models. The results show that GRU performs the best in terms of accurate predictions and biLSTM and LSTM also perform well in predicting the early strokes. By adopting the proposed model, physicians can certainly identify the patients who may likely suffer from strokes in the future. The early detection can assist the doctors for treating the patients on time. Prevention is always better than cure, and timely forecasting of strokes can save many lives.

## 4. Conclusion

In this paper, a framework for identification of bioelectrical signals with the aid of deep learning is proposed that enables the early detection and prediction of stroke disease. The prediction model is capable of learning from offline data and then make predictions on the online data quickly for early detection of strokes. Nowadays, ministrokes/TIA also signifies that the person may get stroke sooner or later. Early detection of signals can certainly assist the physicians to start quick treatments for the prevention of strokes. The damage of stroke is irreversible, and prevention is the only cure for strokes. Hence, this paper is presenting a quick technique based on noninvasive method which uses EEG signals as raw data to train the framework and then to predict whether the person can have stroke in the near future or the signals are normal. The proposed framework uses four different deep learning techniques to check the versatility of the deep neural networks for prediction of strokes, and it is found that all the deep learning techniques can work well for detecting strokes from the biosignals, but GRU and biLSTM outperform the conventional LSTM and FFNN. The accuracy is better with GRU and biLSTM; the prediction error rates are minimal for GRU and biLSTM as compared to LSTM and FFNN. The specificity score obtained by GRU is 0.82, biLSTM is 0.76, LSTM is 0.65, and FFNN is 0.59, whereas the sensitivity score obtained by GRU is 0.94, biLSTM is 0.90, LSTM is 0.85, and FFNN is 0.78. It is a remarkable research outcome that reveals that the stroke could be detected so easily by using the proposed noninvasive framework. In the future, more methods will be considered along with EEG such as ECG and CT scan images for better prediction and prevention of strokes.

## Figures and Tables

**Figure 1:** Architecture diagram of the proposed work.

**Figure 2:** Collection of bioelectrical signals using EEG.

**Figure 3:** Types of EEG waves found in human brain.

**Figure 4:** MAE values obtained by the proposed and other models.

**Figure 5:** RMSE score obtained by the applied algorithms.

**Figure 6:** Presenting MSE values found by applied algorithms.

**Figure 7:** MRE values obtained by diverse techniques in defined iterations.

**Figure 8:** Specificity and sensitivity scores obtained by various techniques.

## Data Availability

The data gathered online can be made available, but offline data which is used for training the module is restricted to share as per the norms of data provider.
